The article "Application of Intelligent Nursing Information System in Emergency Nursing Management" was retracted in 2023. Reasons: signs of a paper mill; suspected computer-generated content; unreliable results or conclusions; lack of ethics approval or compliance.

# Application of Intelligent Nursing Information System in Emergency Nursing Management

**DOI:** 10.1155/2021/3998830

**Published:** 2021-08-04

**Authors:** Qing Li, Yujie Chen

**Affiliations:** Shengjing Hospital of China Medical University, Shenyang, Liaoning 110022, China

## Abstract

This paper is combined with the intelligent nursing information system to build the emergency nursing platform architecture, from the system emergency procedures, system functionality, network environment deployment, and database design aspects of the discussion. Based on hospital information security, the nursing monitoring system of the intelligent nursing information system is constructed to realize network communication, which is clear and intuitive. The intelligent information system is applied to safety control, medical order information, condition information, and information inquiry, which can save working time and complete the rapid transmission and accurate execution of medical order, making the network communication of medical care more quick and convenient and maximizing the overall efficiency. Based on the disordered phenomenon of registration triage, the Relief algorithm is used to classify the aetiology and triage, and the combination of medical advice, information query, and IT technology is optimized, so as to eliminate the phenomenon of round diagnosis, insert number, and improve the medical environment of waiting for diagnosis, taking medicine, examination, and testing. Finally, through the testing of system information security, information traceability, and rapid information query, the problems in nursing management have been basically solved.

## 1. Introduction

The rapid development of computer information technology makes nursing management develop into intelligence gradually. Foreign researchers use Internet technology to connect nursing management to the hospital information network so that medical staff can obtain patients' physical signs data remotely. The nursing management system uses information technology to set various parameters in advance. The system can set various parameters in advance, the system can remind the patient to take medicine on time according to the parameters set, and the collection of the patient's signs' data through the Internet can be sent to the terminal, for doctors and family members to view. The social medical service system in China is not perfect. Most patients go to tertiary hospitals regardless of the severity of their illness, which makes the emergency departments of tertiary hospitals overcrowded. When emergency medical resources are inevitably dispersed to noncritical patients, the ability of the entire emergency medical system to treat critically ill patients will decrease. With the increasing workload of emergency departments, manual statistical data and information will be lost to varying degrees, and the preservation, collection, and analysis of emergency medical data lack norms and efficiency. The lack and lag of emergency information management lead to difficulties in the evaluation, monitoring, and analysis of emergency service process, medical quality, workload, and content. Medical information or medical services of digital, network, and information inaction is referred to by computer science and the modern network communication technology and database technology, for each hospital between patients and hospitals between their respective departments to provide information and management information collection, storage, processing, extraction, and data exchange and satisfy the functional requirements of all authorized users. With the development of wireless information technology, mobile communication technology, and Internet of Things technology, it is possible to effectively preserve and standardize the clinical data of emergency patients through the establishment of an integrated information system before and within the hospital. It has become an urgent problem for the development of the emergency department to strengthen the information construction and the application of nursing management data.

The article "Application of Intelligent Nursing Information System in Emergency Nursing Management" was retracted in 2023. Reasons: signs of a paper mill; suspected computer-generated content; unreliable results or conclusions; lack of ethics approval or compliance.

Ang et al. aimed to better apply the nursing information system to nursing management, so as to promote the change of hospital nursing management mode [1]. Jiang proposed the application effect of emergency triage safety management in emergency nursing, effectively improving nursing satisfaction, reducing the incidence of safety accidents, and enhancing the quality of nursing [2]. Al-Fattah et al. proposed to implement the integration of information system platform, prehospital emergency, hospital emergency department, and other emergency procedures seamless; the sharing of medical information of all patients makes the communication between medical care more accurate and timely, optimizes the emergency work process, significantly shortens the rescue time of patients, and saves lives for patients [3]. Yu et al. proposed an intelligent clinical nursing management information system, which can systematically manage the basic work of nurses, monitor the quality of nursing work in real time, record the work of nursing, evaluate the performance of nursing, and so on, meeting the requirements of nursing management normalization [4]. Li et al. introduced an information zed nursing information system in the outpatient department to reduce the treatment congestion in the outpatient and emergency infusion room, improve patients' satisfaction in the clinical nursing process, and reduce the drug depletion rate and the incidence of nursing complaints and errors [5].

The article "Application of Intelligent Nursing Information System in Emergency Nursing Management" was retracted in 2023. Reasons: signs of a paper mill; suspected computer-generated content; unreliable results or conclusions; lack of ethics approval or compliance.

The application and development of nursing information system in the process of clinical medicine practice, the comprehensive development path and development needs of modern clinical nursing work in China show the characteristics of close correlation that cannot be ignored, and the prosperity and development of modern clinical nursing practice create and provide support and guarantee conditions that cannot be ignored [6]. Sharing the communication data information module with the primary hospital nursing information system can provide active support for the construction and development of the remote nursing expert system [7]. Nursing theoretical knowledge and practical experience can be shared in different regions and different hospitals, and remote nursing practice assistance guidance can be carried out. This is the sharing of advanced nursing practice experience across the country, enabling the comprehensive skills of daily nursing practice work organization at all levels of primary hospitals to continuously improve, thereby providing solid and sufficient experience and supporting conditions for construction and promotion.

## 2. Intelligent Emergency Care System

### 2.1. Intelligent Emergency Procedure

The system software consists of two aspects of database and application software, system database through HIS database related tables, to establish patients primary index, application area table, and orders table, to establish relevant views, and to make nursing system tables associated with HIS data table and data table field be extended, so as to improve the efficiency of the system maintenance and access [8]. The system is developed by using 3-layer B/S architecture. The database is connected by Oracle DBC driver to realize the mutual connection of data. The hospital Intranet enables access to fixed workstations and mobile nursing workstations via the wireless network in the hospital. For other clients such as handheld nursing record terminals, nurse workstations, and mobile ward rounds, the system can be accessed through all compatible browsers except for PDA terminals. The PDA terminal is developed with the template of the Smart Device Cab Project, which can work online or offline. The specific software process is shown in Figure 1.

### 2.2. Basic Architecture of Intelligent Emergency Care

The intelligent emergency centre applies intelligent information technology to the emergency environment with strict real-time requirements. As the intersection of modern information technology and medicine, the intelligent emergency centre has broad development space and practical value. According to the current situation of the low emergency degree in emergency centres and combined with the urgent and hectic characteristics of emergency medical work, an information project was designed and implemented [9]. Based on the hospital network platform, the layout structure, business process, service management, and quality control of outpatient and emergency departments are optimized in an all-round way, so as to alleviate the pain of patients. In this whole process link to develop the corresponding information system, intelligently building this platform, with platform “all-in-one-card” as the core, it runs through the whole process of prehospital appointment, in-hospital reception and treatment, posttreatment inquiry, and evaluation: making an appointment, self-help leading examining, self-help do card, prepaid phone, registering, clinic queuing howl, outpatient doctor workstation, taking medicine denominated in a queue, auxiliary diagnosis department charge confirmation, blood line up your turn, check the line up your turn, inspection result message booking, inspection report self-service printing, mobile infusion, EICU intensive care, patients self-help query, hospital self-help evaluation system, restructuring the medical treatment process with the implementation point deduction mode, changing the traditional medical treatment mode of outpatient department, realizing the complete sharing of business data, the maximum optimization of the medical treatment process, and the quality supervision of the whole process.

The article "Application of Intelligent Nursing Information System in Emergency Nursing Management" was retracted in 2023. Reasons: signs of a paper mill; suspected computer-generated content; unreliable results or conclusions; lack of ethics approval or compliance.

According to the work unit of the emergency centre, the digital system designed eight subsystems, including registration workstation, triage workstation, consulting workstation, emergency room workstation, ICU workstation, doctor workstation in observation ward, nurse workstation in observation ward, infusion room workstation. Registration workstation is to complete the patient's basic information entry and registration. The triage workstation will guide the patient to the corresponding consultation room according to the condition. The clinical workstation completes the treatment of very urgent and critically ill patients. According to the particularity of the work of the emergency room, the functions of the emergency room workstation include the management of access to the department, the treatment of medical orders, the documentation of the course of the disease, and the management of expenses, realizing the automatic valuation of medical orders and the automatic generation of various disposal orders. The ICU workstation system is equipped with a nurse station and doctor station, automatically generating special nursing record sheets, physical sign observation sheets, and other nursing medical documents and automatically completing fluid balance calculation, critical score, and other services. According to the patient's postoperative recovery, the best treatment plan was developed. The system also supports research statistics, providing first-hand information for the development of evidence-based medicine and critical care medicine. Under observation ward medical and nursing workstation system based on computer of HIS ward management pattern, design features, setting up beds, patient access management, orders issued, copying and filling in the inspection sheet, checklists, writing electronic medical records, medicine and nursing information of the input, pricing, cost management, nursing information management, information query, and so forth, realize the automatic valuation of medical orders, automatic generation of all kinds of disposal lists, reduce the number of manual duplicate copies of medical orders, reduce the workload of medical staff, and realize bedside record of patients' condition information. Set up patient emergency treatment information, vital signs' information, and other files. Complete relevant information input and inquiry processing of patients in emergency operating room workstation. According to the work requirements of the infusion room, the system is equipped with infusion sheet management and patient call response management to complete the call, input, query, and processing of the patient infusion sheet; generate infusion bottle label and respond to the patient's call and other functions. The basic mechanism diagram is shown in Figure 2.

The article "Application of Intelligent Nursing Information System in Emergency Nursing Management" was retracted in 2023. Reasons: signs of a paper mill; suspected computer-generated content; unreliable results or conclusions; lack of ethics approval or compliance.

### 2.3. Intelligent Nursing Monitoring System Framework

Client application: an intelligent terminal used by medical staff to edit and consult business data through this application, which is the user's actual operation interface. It is mainly composed of two parts: Android terminal and iPad. Application server: sandwiched between the database server and the client application, it plays the role of data exchange, is responsible for the implementation of the business logic of the whole system, can carry on the security authentication and the system upgrade to the client, has the role of connecting the preceding and the following, and is the core key of the whole system. Part of the application server is made up of mature and functional Microsoft IIS. Database server: the lowest level of the system, mainly composed of the existing information system of the hospital, which provides data and updates. His, LIS, and EMR are its main components. The monitoring framework is shown in Figure 3.

### 2.4. Intelligent Nursing Function

The intelligent nursing system is that nurses use mobile intelligent terminals to scan the barcode of patients' wristbands, accurately identify the identity of patients, input vital signs beside the patient's bed, and write the condition observation, so as to reduce paper transcribing, reduce workload, and improve the accuracy and timeliness of nursing work [10]. Nurses scan the barcode of medicines and check patients' wristbands through handheld smart terminals to avoid medical errors. At the same time, the closed-loop implementation of the doctor's order is achieved, and the traceability problem of the infusion and drug is realized. The mobile nursing subsystem not only ensures the safety of patient diagnosis and treatment but also evaluates the performance of nursing work, guarantees the safety of patients' clinical nursing, improves the nursing level, and normalizes nursing behaviour [11]. The functional requirements of the intelligent nursing system are shown in Figure 4.

  Bulletin board: this interface displays the basic information of the ward of the hospital, such as the number of patients in the ward, the grade of nursing, and the information of critical patients. The key point records at work should be viewed and edited by all nurses in the ward, and the head nurse needs to manage; the ward nurses work in some requirements of the record.
  Execution of medical orders: the mobile nursing subsystem is mainly to execute the clinical medical orders and complete the closed-loop operation of medical orders. Entering the doctor's order execution window and scanning the barcode on the patient's wristband, you can view the doctor's order items that the patient has executed and the doctor's order items to be executed. The patient's infusion bottle sticker, drug package barcode, and test tube barcode can be scanned again to complete the closed-loop execution of infusion and medication and test doctor's orders. The barcode of patients' wristbands, drugs, infusion, and test specimens can be matched one-to-one, which not only realizes the traceability of medical orders but also effectively fills the last ten meters of medical workstations and patients' beds.
  Nursing evaluation: within 24 hours of admission, nurses need to conduct admission nursing evaluation, fall bed evaluation, and pressure sores nursing evaluation on patients through mobile handheld terminals, so as to understand the basic situation of patients, determine the nursing level of patients, reduce a large number of nurses to copy labour, and improve nursing efficiency.
  Nursing records: all nursing services received by patients should be recorded through intelligent terminals, nursing data should be saved, patient nursing data should be summarized, effective management of nurse nursing services can be realized, service quality can be improved, and patient satisfaction can be promoted.
  Vital signs: the nurse can connect the internal network of the hospital through the intelligent handheld terminal and record the patient's temperature, pulse, respiratory frequency, frequency of urine, and faces beside the patient's bed, which will be synchronized to the hospital database server and sent to the doctor in time to provide a medical diagnosis. At the same time, the system can carry out the batch entry of vital signs and accurate and efficient entry of patients' nursing indicators.
  Voice call: when the infusion is about to end in the ward, the patient's family members or patients themselves need to go to the nurse station to remind the nurse that the infusion is about to run out, and the needle can be pulled out or the bottle can be changed. In practice, the information that “infusion is about to end” cannot be conveyed to the treating nurse due to various conditions of the patient. It not only affects the treatment of patients but also has life-threatening risks, and the timeliness of artificial oral replacement cannot be guaranteed. Through the intelligent nursing system, a direct voice call can be made to the current treatment nurse in the ward, informing the responsible nurse in the first time, so that patients can run fewer errands and much information.
  Thermometer distribution: at this stage, the patient's temperature is mainly measured through a mercury thermometer, and then the nurse takes back the thermometer and records it. Due to the large number of rooms and patients in the ward, it is often not possible to clearly record the distribution of thermometers. The intelligent nursing system has the function of thermometer management, which records the distribution of the thermometer and reminds the nurse to recover the thermometer after the end of the measurement time, so as to achieve accurate management.
  Ward patrol: according to the time required by the standard of graded nursing, the nurse needs to patrol the ward according to the condition and needs of special patients. The mobile nursing system adopts a ward inspection interface, which is convenient for nurses to scan patients' wristbands, conduct ward inspections, record inspection data, and collect them at the end of the month, so as to realize the assessment of nursing quality.

The article "Application of Intelligent Nursing Information System in Emergency Nursing Management" was retracted in 2023. Reasons: signs of a paper mill; suspected computer-generated content; unreliable results or conclusions; lack of ethics approval or compliance.

### 2.5. Multisystem Integration

Integration is to integrate several small systems with different functions into a large system with multiple functions by using systems engineering theory, so as to give full play to the comprehensive efficiency of the large system [12]. Intelligent emergency centre is an intelligent system with a complex structure that integrates HIS, LIS, PACS, critical care information system, emergency information system, and other functions related to emergency treatment. The system will be doctors and nurses operation process; inspection, application for inspection, and return of results; handling of charge accounting; and department management and other links into the computer management system, to replace the flow of people with information flow, to realize the emergency centre of the flow of people, logistics, capital flow, and other information implementation of decentralized collection, unified management, centralized use, and all the automated mode of sharing, to provide a fast navigation device or interface for medical staff. It is the emphases and difficulties of the research to enable doctors to switch quickly among various systems and apply various information synthetically. System integration is shown in Figure 5.

### 2.6. System Network Design

In the construction of the mobile medical system, the wireless network is the top priority. Only a scientific overall structure of the wireless network can achieve stable and high-speed data transmission. The ward in the hospital is different from the general conference venue. There are many rooms in the hospital. The room area is large, the walls are thick, the corridor of the department is long and narrow, and there are various cables such as oxygen, circuit, and communication above the ceiling, and the environment is complex. In view of the above special environment and the actual situation of the hospital, wireless controller, wireless switch, and wireless access point are adopted to build the hospital wireless network [13]. The topology of the wireless network is shown in Figure 6.

## 3. Application of the Intelligent Nursing Information System

### 3.1. Application and Management of the Intelligent Protest and Triage System

The automatic classification of quantified triage indicators and region-oriented intelligent triage system are based on the quantifiable triage standard system of emergency reexamination and triage, and the intelligent software of emergency reexamination and triage is developed by using computer technology to realize computer-aided reexamination and triage [14]. The intelligent triage system for patients' disease classification mainly takes the symptoms of body parts as the evaluation guide; inputs the patient's name, age, vital signs parameters, pain score, adjustment parameters, and so on the computer; and automatically generates the patient's condition grade. At the same time, a printer is connected to print out the patient's information and grade on red, yellow, and green printed paper and affixed to the patient's medical record. The principle of disease classification and treatment time in our hospital is as follows: red refers to Grade 1 resuscitation or endangered patients, and patients are directly sent to the emergency room in the red zone. The first-grade critically ill patients were rescued immediately and treated within 15 minutes in the red zone or the yellow zone. Level 2 emergency patients: according to the condition, emergency arrangement of priority diagnosis and treatment is generally done within 30 minutes of emergency treatment in the yellow area. Level 3 nonemergency patients are treated sequentially in the green area and treated within 2 hours.

The article "Application of Intelligent Nursing Information System in Emergency Nursing Management" was retracted in 2023. Reasons: signs of a paper mill; suspected computer-generated content; unreliable results or conclusions; lack of ethics approval or compliance.

The triage desk is equipped with an auxiliary triage system connected to command platform, which releases the general information of the next emergency patient on the LED display terminal in advance, including gender, age, main illness, departure place, and approximate arrival time; makes full preparations for supplies; and informs the doctor in advance of the layout and equipment of 1 division. At the time of developing the intelligent triage system, the environment of the emergency room was modified to match its function. Three colours of red, yellow, and green represent the three areas in the transformed emergency department, and the background decoration and medical signs in each area are corresponding colours. The red area is the emergency room, the yellow area is the emergency treatment area, adjacent to the emergency room, and the green area is the general treatment area. In addition, red, yellow, and green landmarks are adopted in the emergency area, and the arrow guiding function is clear at a distance. The emergency hall provides TV and wireless network and other services to improve details and humanized services, which to some extent reduces the anxious state of patients waiting for treatment.

Division nursing human resources allocation and management personnel management is mainly for the yellow area, the green area, and the prediagnosis table. Since the general diagnosis and treatment is divided into yellow area and green area, one more itinerant nurse is added to carry out treatment and health education and other services for emergency patients in the yellow area. The other nurse is mainly responsible for the order of the rooms in the yellow area and the green area and the coordination of patient diversion. Due to the use of the new intelligent system, the workload of prediagnosis increased. Two nurses were assigned to the post and the admission system of prediagnosis nurses was established. Only those with certain working experience, clear thinking, and qualified training of the new system could take the post. The prediagnosis nurse makes the correct disease classification, communicates with the itinerant nurse in time, and plays a guiding role in the patient's regional consultation.

The article "Application of Intelligent Nursing Information System in Emergency Nursing Management" was retracted in 2023. Reasons: signs of a paper mill; suspected computer-generated content; unreliable results or conclusions; lack of ethics approval or compliance.

### 3.2. Intelligent Nursing Safety Control Application

Patient safety control is primarily concerned with problematic areas of health care, particularly the identification of patients during the administration of drugs, transfusions, or blood products; the drawing of blood or the testing of other clinical specimens; or the delivery of treatment or procedures. The hospital's compliance with patient safety objectives is regarded as an independent decision item in the review and decision-making process, and the one-vote veto system is implemented. It can be seen that patient safety plays a very important role in the quality of hospital medical service.

At present, barcode technology has been widely used in the system, outpatient and emergency mobile infusion management system, prescription dispensing subsystem, etc., providing a simple and convenient management approach for the safety control of outpatient and emergency patients. A barcode is a mark that expresses a group of information by arranging multiple black bars and blanks with different widths according to certain coding rules [15]. The bar is the part that is less reflective of light, and the empty is the part that is more reflective of light. Barcode technology is born along with the development and application of computer and information technology. It can be converted into binary or decimal information which can be recognized by the computer. It is a new technology integrating coding, printing, identification, and data acquisition and processing. In the process of medical service, the barcode can be used as the identification information and scanned by the scanning gun to realize the rapid extraction of the corresponding patient information from the database of the computer system. The hospital tests equipment to achieve all online.

The whole inspection process includes barcode label printing, barcode specimen identification processing, report feedback transmission, and self-service query and printing of clinical departments and outpatient and emergency patients. Barcode technology plays an important role in the diagnosis and treatment of outpatient and emergency infusion. In the past, the outpatient and emergency infusion is manually checked by the nurse, the liquid, and the filling of drugs. The nurse checks again and again, which is inefficient and risky. The outpatient mobile infusion management system automatically generates the patient's barcode information by computer and automatically prints two sets of infusion cards with identical information, including the patient's name, gender, age, drug dose, concentration, drip count, time of treatment, and other information. One is given to the patient for scanning at the time of injection, and the other is affixed to the pouch. Before the injection, the nurse uses a handheld computer to scan the barcode of the infusion card on the soft infusion bag. An electronic voice system automatically calls the number, and the patient hears the call and arrives at the puncture table. If the patient's line does not match the barcode of the fluid, the computer will send an alarm to remind the patient not to inject. After the infusion, the palm computer scanning, the patient's total bag of infusion, each bag of drug type, specific time, and infusion process can be clear at a distance, before pulling out the needle to understand the patient's treatment effect, after the confirmation of the end of treatment and then pulling out the needle. The use of barcode can effectively identify the identity of patients and drugs in both directions, which adds a safe defence line for outpatient and emergency infusion management. While optimizing the traditional workflow, it reduces the labour intensity of nurses and improves their work efficiency. The infusion card and bottle label are automatically printed to avoid the hidden danger caused by unclear handwriting by hand, check the infusion drugs with patients, and implement the system of three checks and eight pairs into the monitoring state to ensure the safety of patients' medication and treatment.

The article "Application of Intelligent Nursing Information System in Emergency Nursing Management" was retracted in 2023. Reasons: signs of a paper mill; suspected computer-generated content; unreliable results or conclusions; lack of ethics approval or compliance.

### 3.3. Intelligent Nursing Medical Advice Information Application

After the nurse scans the barcode of the patient's wristband through the intelligent terminal, the patient is identified and the detailed information of the patient is displayed, as well as the content of the doctor's order. According to the type of the doctor's order, the label is divided into infusion book, treatment book, medication book, doctor's order book, new start, and new stop. The nurse can directly click the execute button on the doctor's order information to execute or confirm the execution by scanning the outer package of the drug, the infusion bottle sticker, and the barcode on the test tube. Meanwhile, the system automatically records the executor and the execution time [16]. The diagram of the medical order processing module is shown in Figure 7.

### 3.4. Intelligent Nursing Letter Observation Application

By observing the patient's mental state, consciousness, and mobility, the nurse writes the nursing assessment sheet, the risk assessment sheet of falling on the bed, and the admission assessment sheet [17]. At the same time, nurses can record nursing and nursing measures in the intelligent terminal and can also save the written content as a template and view the historical nursing data. The module diagram of disease observation is shown in Figure 8.

### 3.5. Integrated Query Information Module Application

After the nurse logs in the system, the patient is displayed in the form of a label, which contains the patient's name, gender, age, bed number and other basic information. After clicking the label, the detailed information of the patient can be viewed, including diagnostic information, nursing level, allergy drugs, attending physician, and other information. The nurse can also click on the patient's label to see the patient's medical record and examination report, as well as the patient's expense information: advance payment, expense details, and account balance. The comprehensive query module is shown in Figure 9.

## 4. Debugging and Testing of the Intelligent Nursing System

### 4.1. Information System Selection Method

Relief algorithm was first proposed by Kara, aiming at two classification problems, and its theoretical basis is as follows: a good feature should make the similar sample of the nearest neighbour characteristic values between the same or similar, and the nearest neighbour value differences between the different classes of samples or difference are very big, therefore giving each feature corresponding weights for sorting; the greater the weight of characteristic, the stronger the feature classification ability; on the contrary, the feature classification ability is weak. By setting the feature weight threshold or the number of feature subsets, the corresponding feature selection can be carried out, and the feature can be evaluated according to the feature's ability to distinguish the close samples. The main idea behind Relief's algorithm is that good features should keep samples of the same class close and samples of different classes away. Assume that the interval is defined as the maximum distance that the decision surface can move without changing the sample classification, which can be expressed as

(1) $$\begin{array}{c} \phi =11\;\times \;\left(\left|x-y_{x}\right|-\left|x-h_{x}\right|\right), \end{array}$$

where *Y*_*x*_ means similar to *x* and *h*_*x*_ with *x* means nonhomogeneous nearest neighbour.

The article "Application of Intelligent Nursing Information System in Emergency Nursing Management" was retracted in 2023. Reasons: signs of a paper mill; suspected computer-generated content; unreliable results or conclusions; lack of ethics approval or compliance.

The weight of the update attribute *P* of sample *X* can be expressed as

(2) $$\begin{array}{c} W_{p}^{i+1}=W_{p}^{i}-f\left\{p,x,H_{j}\left(x\right)\right\}+\frac{P\left(x\right)}{1-P\left(x\right)}\times f\left\{p,x,H_{j}\left(x\right)\right\}+m. \end{array}$$

Koromiko extended the Relief algorithm to get the Relief algorithm, which can be applied to multiple sample cases. When dealing with multiclass problems, the Relief algorithm does not uniformly select the nearest neighbour samples from all sample sets of different classes but selects the nearest neighbour samples from each sample set of different classes and selects *k* nearest neighbour samples. The weight update formula is

(3) $$\begin{array}{c} W_{p}^{i+1}=W_{p}^{i}-\sum_{j=1}^{k}f\left\{p,x,H_{j}\left(x\right)\right\}+\sum \frac{P\left(x\right)}{1-P\left(x\right)}\sum_{j=1}^{k}f\left\{p,x,H_{j}\left(x\right)\right\}+m\times k. \end{array}$$

Artificial Fish Swarms Algorithm is a swarm intelligence optimization algorithm based on fish swarm behaviour proposed by domestic scholars Ian Jixi and Li Xiao lei et al. According to the bionic characteristics of fish swarm, it simulates foraging, clustering, and tailgating behaviours of fish swarm by constructing artificial fish [18], so as to realize optimization. Artificial fish include the following behaviours. Foraging behaviour: assume that the current state of the artificial fish is *Xi*, and select a state *x* within its field of vision at random. If *Yi* < *I*, it will move further in this direction; otherwise, it will move one step at random. If the constraint is not satisfied, cut it out:

(4) $$\begin{array}{c} \left(\begin{array}{ccc} x_{j} & \ldots & y_{j}\\ \vdots & \ddots & \vdots \\ y_{\mathrm{jn}} & \cdots & x_{\mathrm{jn}} \end{array}\right). \end{array}$$

### 4.2. Intelligent Triage Disease Grading Factors

Patients with acute and critical illness are mainly aged, and by referring to the previous data of researchers, three levels of proportions are summarized, among which patients with grade over 60 years old account for 58.45% of the total number of patients, and patients with grade A only account for 41.55%. It can be seen that the elderly population is typical potential acute patients, and the elderly patients with grade A are the focus group in the dynamic triage process.

The correlation of blood pressure indexes in patients with II grade critical illness was gradually enhanced with the increase of blood pressure, suggesting that blood pressure was of great significance in the recognition of the disease in patients with the normal grade, while there was no significant correlation in patients with the mild or moderate grade. The possible reasons for the correlation were as follows: III grade acute patients with more acute symptoms, but the vital signs are stable, although there is a risk of deterioration, but there is no risk of life-threatening or disability, so the abnormal blood pressure exposure is not obvious; IV grade nonemergency patients mostly have no acute symptoms, and almost no exposure to abnormal blood pressure, or after brief exposure, it can be relieved and disappear after rest.

The article "Application of Intelligent Nursing Information System in Emergency Nursing Management" was retracted in 2023. Reasons: signs of a paper mill; suspected computer-generated content; unreliable results or conclusions; lack of ethics approval or compliance.

Breathing and blood oxygen saturation index reaction is a more sensitive index for the human body, breathing >20 times/min, the total number of I∼III levels accounted for 89%, and 60.98% were III level; therefore the postoperative respiratory management of critically ill patients directly affects the survival and quality of patients, which is acute and potentially dangerous. Paying close attention to changes in breathing is important for early recognition and correct treatment.

On the basis of preliminary construction of emergency patients nursing difficulty evaluation index system, the results summed up four categories of influencing factors: patient factor, nurse factor, organizational factor, and nursing equipment condition factor. Among the patient factors, 7 factors were extracted, including age, severity of disease, self-care ability, mental and psychological status, social support system, compliance, and expectation [19].

Patient expectation refers to the degree to which patients place their expectations and wishes on medical institutions before treatment, which is mainly reflected in treatment effect, treatment cost, medical service quality, length of hospital stay, and pain in the process of diagnosis and treatment. The influencing factors include individual needs of patients, commitment of medical institutions, medical experience of patients, and severity of diseases [20]. The first-level indicators are broken down as follows: the general condition of patients covers the age and complications of patients. Severity of disease in emergency patients, self-care ability: according to the industry recommended standard published by the National Health and Family Planning Commission Barthes Index Evaluation Table, the evaluation can be divided into four grades, which are, respectively, heavy dependence, moderate dependence, mild dependence, and complete self-care. Mental health status: the Hospital Anxiety and Depression Scale is a self-rating scale [21], including 2 subscales of anxiety and depression, respectively, for 7 questions of anxiety (A) and depression (D). 0–7 are asymptomatic; 8–10 are suspicious. 11∼21 categories definitely have anxiety. Social and economic status: social and economic status is mainly evaluated by three indicators: social support, economic income, and education level. Compliance: observe the patient's compliance to treatment, nursing, and examination and comprehensively evaluate the patient's overall compliance by asking the patient's doctor in charge and the responsible nurse, which can be divided into five grades: very cooperative, cooperative, basic cooperative, noncooperative, and very noncooperative.

The article "Application of Intelligent Nursing Information System in Emergency Nursing Management" was retracted in 2023. Reasons: signs of a paper mill; suspected computer-generated content; unreliable results or conclusions; lack of ethics approval or compliance.

### 4.3. Test Process and Results

In the completion of the design and coding of intelligent nursing information system, in order to ensure that the software shows fatal functional errors, improve the reliability and efficiency of the implementation of the software. Software validation is required according to software functional requirements. When testing the software, make sure you can deploy the appropriate operating system to the business server and install the basic operation profile and execution file.

In this paper, 20 emergency patients were randomly selected and 5 outstanding nursing staff were selected to complete the basic operation, statistical function, and operational function tests of the software functional modules, and the test results of the functional modules were collected and recorded. The basic operation tests are shown in Table 1.

Ten emergency patients were selected for the test, and the basic operation tests of inquiry, physical sign entry, drug dispensing, nuclear drug, patrol, and nursing records were recorded, respectively. The test results are shown in Figure 10.

In order to verify the reliability of the statistical function of the intelligent emergency information system, the beds, workload, execution status, and reminder of the emergency department of a simulated hospital for one week were tested and entered into the system. The test results are shown in Figure 11.

The sensitivity of the intelligent nursing system to the screening of patients in the emergency was tested, and 20 emergency patients were randomly selected to enter the sign information. The sensitivity is shown in Figure 12.

The basic operation test in this paper mainly includes inquiry, physical sign entry, drug dispensing, nuclear drug, patrol, and nursing record test. The passing rate of basic operation test and system function test of the intelligent nursing system is more than 94%. Simulating the intelligent nursing system and summarizing the test data, the sensitivity of emergency patient screening was 82.22%, and the predictive index was 85.82%, but 90% are not ideal; it may be related to the small sample size in this study; I and II patients only accounted for 25% of the total; the emergency cancer accounts for about 75% therefore, the specific degree as an important evaluation index system, namely, the identification capability of the emergency patients. Calculating system specificity through artificial fish swarm algorithm, the specificity was 94.67%, and the prediction index for nonemergency patients was 91.03%, indicating that the system had a good effect on objective and quantitative identification of nonemergency patients. In the case of limited time and emergency resources, potential risk patients could be found, so as to ensure the safety of emergency patients and assist triage nurses in making decisions on a reasonable allocation of emergency resources.

The article "Application of Intelligent Nursing Information System in Emergency Nursing Management" was retracted in 2023. Reasons: signs of a paper mill; suspected computer-generated content; unreliable results or conclusions; lack of ethics approval or compliance.

## 5. Conclusion

In this paper, an intelligent information zed nursing system is constructed to realize the information sharing in the whole domain, and intelligent auxiliary diagnosis and treatment information is provided to facilitate nursing inquiries of diagnosis and treatment information, which is of great help to patients' follow-up medical activities such as condition analysis, medical history grasp and supplement, and disease diagnosis. The data information stored completely through barcode intelligent information makes it more convenient for medical staff to collect cases and carry out nursing management. At the same time, nursing management online and bar code information collection, without manual transcription and triage, make nursing management faster, more accurate, and more reliable. This shortens the time for emergency nurses to complete the special care record form and effectively reduces the workload of medical staff. It maximizes the integration and utilization of quality-related information through emergency care terminal services.

## Figures and Tables

**Figure 1:** Intelligent emergency procedure.

**Figure 2:** Basic architecture of intelligent emergency care.

**Figure 3:** Basic architecture of intelligent nursing monitoring.

**Figure 4:** Intelligent nursing function.

**Figure 5:** System integration diagram.

**Figure 6:** Wireless network topology.

**Figure 7:** Medical order processing module diagram.

**Figure 8:** Module diagram of disease observation.

**Figure 9:** Comprehensive query module diagram.

**Figure 10:** Statistical chart of nurses' basic operation test.

**Figure 11:** Statistical functional test diagrams.

**Figure 12:** Intelligent recognition level sensitivity map.

**Table 1:** The basic operation tests.

Test project	The test operation	Test result
Inquire	Scan the patient's wristband	Display basic patient information
Signs of entry	Enter the signs and click save	Save record results
Dispense medicines	Click on the dispensing	Prepare medicine as prescribed
Nuclear medicine	Scan the barcode of the infusion	The barcode is the same as the patient
Walk around	Inspect patient information after matching	Record client information after tour
Nursing record	Click on basic care	Display basic care information

The article "Application of Intelligent Nursing Information System in Emergency Nursing Management" was retracted in 2023. Reasons: signs of a paper mill; suspected computer-generated content; unreliable results or conclusions; lack of ethics approval or compliance.

## Data Availability

Relevant data are available upon request to all authors.
